RETRACTED

# Effects of Pelvic Floor Muscle Training Combined with Estriol on Pelvic Floor Dysfunction after Total Hysterectomy Applied in Perimenopause

**DOI:** 10.1155/2022/6962542

**Published:** 2022-07-18

**Authors:** Jichao Jin, Minyuan Wang

**Affiliations:** Department of Obstetrics and Gynecology, The First People's Hospital of Wenling, Taizhou, Zhejiang 317500, China

## Abstract

**Objective:**

Total hysterectomy (TH) is becoming more and more common in clinical practice, and many patients suffer from postoperative complications such as pelvic floor dysfunction (PFD). How to prevent and treat PFD is an important part of the current clinical work, and it is important to improve patients' postoperative quality of life. This study was to investigate the effect of pelvic floor muscle training (PFMT) combined with estriol on PFD after TH in perimenopause.

**Methods:**

Totally, 95 patients who developed PFD receiving TH in our hospital between January 2020 and June 2021 were selected. They were randomly divided into a PFMT+ET (estriol therapy) group (*n* = 49) and CT group (conventional treatment, *n* = 46). After treatment, the two groups were compared in terms of pelvic floor muscle tension (systolic pressure and resting pressure of the vagina), female sexual function index (pain, satisfaction, orgasm, sexual arousal, sexual desire, and lubrication), and the degree of PFD (persistent time of vaginal muscle contraction, 1-hour pad test, residual urine volume, and frequency of urinary incontinence).

**Results:**

After 4 months of treatment, vaginal systolic pressure and resting pressure were significantly increased in both groups, with higher levels in the PFMT+ET group. Also, the improvement in female sexual function index score and persistent time of vaginal muscle contraction was observed to be greater in the PFMT+ET group than in the CT group. Additionally, PFMT combined with estriol resulted in lower levels of urinary leakage in the 1-hour pad test, residual urine volume, and frequency of urinary incontinence.

**Conclusions:**

The postoperative intervention of PFMT combined with estriol in perimenopausal patients with TH can significantly improve vaginal muscle contraction, improve the quality of sexual life, and reduce the degree of PFD, which has a good application prospect.

## 1. Introduction

Currently, the probability of receiving total hysterectomy (TH) has climbed up [1]. As a common gynecological procedure, TH is often applied to cure diseases that require the removal of the uterus such as hysteromyoma, uterine adenomyoma, endometrial hyperplasia, and dysfunctional uterine bleeding. However, this surgery may cause damage to the pelvic floor structure, pelvic nerves, and pelvic organs, triggering common complications such as pelvic floor dysfunction (PFD) [2, 3]. Studies have shown that the incidence of PFD after TH is approximately 17%, which has been found to be significantly related to age-induced pelvic floor muscle atrophy, times to give birth, obesity, and postoperative pelvic floor muscle training (PFMT) [4]. Common manifestations of PFD mainly include bladder dysfunction (bladder paralysis, urinary retention, and urinary incontinence), sexual dysfunction (decreased libido, vaginal dryness, dyspareunia, and loss of orgasm), and defecatory dysfunction (constipation), seriously affecting the quality of life and mental health of patients [5]. Therefore, the treatment of PFD after TH has become an important issue that needs to be addressed urgently.

RETRACTED

Intervention targeting the pelvic floor following TH is an important measure to prevent PFD. At present, the common treatments for the recovery of pelvic floor function after TH mainly encompass PFMT, pelvic floor muscle electrical stimulation, bladder training, *α*-adrenergic agonist, and topical vagina hormone therapy. Such nonsurgical treatments improve the symptoms of 30%-60% of patients [6]. Pugsley et al. believe that a conscious effort to train the pelvic floor muscle after surgery can also help to prevent urinary retention and urinary incontinence and to improve PFD [7]. Radzimińska et al. demonstrated that PFMT can treat female urinary incontinence and improve quality of life [8]. In addition, when adopted after TH, estriol can cut down the rate of infection, maintain the balance of vaginal bacteria, promote wound healing, and facilitate the recovery of PFD [9]. Estriol is a natural estrogen mainly present in urine. Its clinical application can improve stump healing and kill vaginal pathogens [10]. However, vaginal estrogen therapy alone has a short-term improvement in PFD symptoms in perimenopausal women [11]. The combination of pharmacological treatment and physiotherapy is a better intervention for patients with PFD and may be more effective than single medication, physiotherapy, or rehabilitation training [12]. However, there is a lack of reports in this field. Therefore, in order to find better treatment options, the present study was conducted to observe the therapeutic effects of neuromuscular electrical stimulation and estriol intervention on pelvic floor muscle tone, female sexual function index, and degree of pelvic floor muscle dysfunction in patients with perimenopausal total hysterectomy, so as to analyze the effects of intervention on pelvic floor muscle dysfunction in patients.

## 2. Materials and Methods

### 2.1. Patient Data

A total of 95 patients who developed PFD after receiving TH in our hospital between January 2020 and June 2021 were selected. They were then randomly separated into a PLMT+ET group (pelvic floor muscle training+estriol therapy, *n* = 49) and CT group (conventional treatment, *n* = 46) using the random number table. Inclusion criteria were as follows: (1) perimenopausal women aged 40-55 had sexual experience; (2) patients underwent laparoscopic TH due to benign uterine diseases and were diagnosed with PFD according to the criteria specified in *Advance of Diagnosis and Management of Female Pelvic Floor Dysfunctional Disease* [9] after surgery; (3) there were no other postoperative complications or minor complications that did not affect this study and could be recovered after appropriate interventions; and (4) patients and their families knew and understood this study, complied with the grouping and corresponding treatment, and all signed the informed consent form. Exclusion criteria were as follows: (1) patients with low compliance; (2) patients with a history of PFD caused by other reasons or pelvic floor surgery; (3) patients with urinary system diseases and severe diseases of the heart, liver, kidney, or other vital organs or patients complicated with diabetes or obesity; and (4) patients with asthma, intractable constipation, or malignant tumors. The informed consent form has been signed by patients and their families. (5) The patient was sexually inactive for a long time before the operation and had sex less than once a month. This study was approved by the Ethics Committee of the First People's Hospital of Wenling (no. WMY202009) and in conformity with the Declaration of Helsinki.

RETRACTED

### 2.2. Treatment Methods

In the CT group, corresponding conventional drugs (including anti-infection, regulation of water-electrolyte balance, and symptomatic support therapy) and nursing interventions were given after surgery according to the patient's condition. The ureteral catheter was indwelled for 4 days. In the first 2 days, the catheter was in an open state. On the 3^rd^ day, bladder muscles were exercised by opening the catheter at an interval of 2-3 hours or opening it when there was a desire to urinate and then closing it. This training was in an intermittent and repetitive manner. On the 4^th^ day, the catheter was removed. At the same time, electrical stimulation biofeedback therapy was also performed twice a week for 30 min each with a frequency of 5-50 Hz, at an intensity of 8-20 mA, for 4 months as a course of treatment. During treatment, routine care of the vaginal orifice, urethra, and other parts was maintained. Besides, timely and individualized psychological counseling was also available for patients suffering from anxiety, depression, and other adverse psychological conditions. The condition of patients was closely observed throughout the course.

RETRACTED

In the PFMT+ET group, estriol vaginal cream (0.5 g/day, H20170005, Organon (Ireland) Ltd.) and targeted PFMT were applied in addition to routine nursing. To be specific, there were four steps of PFMT. Firstly, patients were placed in a supine position with legs slightly bending and spreading, and the anal sphincter was forcefully contracted to imitate holding urine for 5 s and then slowly relaxed. Secondly, the patient remains in the supine position with the legs alternately elevated to 90° and then slowly lowers the legs. Thirdly, patients changed to a kneeling position and elevated their legs backwards alternately and then slowly put down the legs. Fourthly, patients returned to a supine position with feet flat on the bed and knees bent and slowly raise the back and buttocks and then slowly put them down. Each step was repeated for 15 min, twice daily (morning and evening), and a course of treatment lasted for 4 months.

### 2.3. Outcome Measures

The two groups were compared at 1 week and 4 months after surgery in terms of pelvic floor muscle tension, female sexual function index (FSFI), and degree of PFD.

Pelvic floor muscle tension was quantified as follows. A pressure balloon was placed in the vagina. Later, vaginal systolic pressure (VSP) and vaginal resting pressure (VRP) were measured after inflating 15 ml of gas.

FSFI included 6 items (pain, satisfaction, orgasm, lubrication, sexual arousal, and sexual desire) and had a total score of 36 points. The higher the index, the better the sexual life. A score > 26.55 indicated the absence of female sexual dysfunction.

The degree of PFD was evaluated by persistent time of vaginal muscle contraction, 1-hour pad test, residual urine volume, and frequency of urinary incontinence.

### 2.4. Statistical Analysis

SPSS 24.0 was used for data analysis. The measurement data were expressed as mean ± standard deviation (SD), and the independent sample *t*-test was used for comparison between groups and the paired *t*-test was used for comparison within groups before and after the intervention. Enumeration data were expressed as frequency (*n*) or rate (%), and the chi-square test (*χ*^2^) was used for statistical analysis. When *P* < 0.05, the difference was considered significant.

## 3. Results

### 3.1. General Information of Patients

A total of 95 patients, aged 43-55 years, were randomly divided into the PFMT+ET group and the CT group. There were no significant differences between the two groups in age, number of deliveries, and primary disease before treatment, indicating that the two groups were comparable (*P* > 0.05, Table 1).

RETRACTED

### 3.2. Efficacy of the Two Treatments on Pelvic Floor Muscle Tension

The effects of PFMT combined with estriol on postoperative pelvic floor muscle tension were probed into in this part. According to the results, there was no significant difference in VSP and VRP before treatment in the two groups, indicating comparability (*P* > 0.05). After treatment, VSP and VRP in both groups were significantly higher than those before treatment (*P* < 0.05), suggesting that both therapies can effectively restore pelvic floor muscle tension, but the efficacy of the combined treatment was superior to that of the conventional treatment (Table 2).

### 3.3. Comparison of Sexual Function Indices between the Two Groups of Women before and after Intervention

There were no significant differences in pain, satisfaction, orgasm, arousal, lubrication, sexual desire, and total score of sexual function indices between the two groups of female patients before the intervention (all *P* > 0.05). In contrast, after the intervention, these indices were significantly higher than those before the intervention in the same group (all *P* < 0.05). And after the intervention, except for lubrication, there was no significant difference between the two groups. All other indices were significantly higher in the PFMT+ET group than in the CT group (all *P* < 0.05) (Table 3).

### 3.4. Comparison of the Degree of Pelvic Floor Muscle Dysfunction between the Two Groups after the Intervention

The duration of vaginal muscle contraction, 1-hour pad test volume, residual urine volume, and frequency of incontinence were not significantly different between the two groups before the intervention (all *P* > 0.05). After the intervention, the duration of vaginal muscle contraction was significantly higher than that before the intervention, while 1-hour pad test volume, residual urine volume, and frequency of incontinence were significantly lower (all *P* < 0.05). In addition, all of these indicators were significantly improved in the PFMT+ET group after the intervention compared with the CT group (all *P* < 0.05) (Table 4).

## 4. Discussion

In recent years, the incidence of pelvic diseases in perimenopausal women has seen an increase. Among the diseases, the incidence of PFD after TH is also high, and it will seriously affect the physical and mental health and reduce life quality of patients without timely intervention [4]. PFD can further cause urinary incontinence, pain, and organ prolapse, and these complications can increase the incidence of infection, pressure sores, and venous thrombosis, which can be life-threatening in severe cases [13]. Therefore, the treatment of PFD after TH needs to be urgently addressed.

RETRACTED

Studies have confirmed that PFMT with or without adjunctive modalities can improve or cure urinary incontinence, fecal incontinence, perinatal and postpartum pelvic floor dysfunction, and sexual dysfunction [14]. In this study, the routine PFMT was enriched and optimized according to the patients' condition, and the patients were supervised to complete the required amount of exercises on time. The improved PFMT has the advantages of noninvasiveness and easy operation and can obtain better rehabilitation effects. We found that pelvic floor muscle tension including VSP and VRP was restored in the two groups, but the therapeutic effect in the PFMT+ET group was proven better. Our findings were consistent with the study by Jiang and Rong [15] reporting that pelvic floor muscle training combined with biofeedback therapy could reduce the occurrence of PFD after TH.

In addition, PFMT combined with estriol was more effective than conventional treatment in improving the female sexual function index in terms of pain, satisfaction, orgasm, sexual arousal, and sexual desire except for lubrication. PFMT combined with estriol also achieved better results of PFD indicators such as persistent time of vaginal muscle contraction, urinary leakage in 1-hour pad test, residual urine volume, and frequency of urinary incontinence, which concurred with the findings proposed by Ye et al. [16]. Possible reasons behind the above results of the combined treatment may be that the regular and effective PFMT after surgery helps patients to complete contraction and relaxation of pelvic floor and bladder muscles, thus promoting pelvic floor blood circulation, metabolism of inflammatory factors, and repair process of pelvic nerves.

Although some meaningful observations were reported, there are still some shortcomings that deserve to be described. First, only 95 cases were investigated in this study, which is a small sample size. Second, the lack of follow-up records does not allow for a valid assessment of the long-term treatment effects of PFMT combined with estradiol. Therefore, larger trials and longer follow-up periods are necessary. Additionally, it is worth noting that patients need to pay attention to gradual and measured PFMT; otherwise, the training intensity exceeds the body's tolerance and may lead to damage to the body. And one should also pay attention to the dosage of estriol when administering medication; otherwise, the body may consume too much estriol, which may lead to disruption of the internal environment and disruption of the hormonal balance in the body, leading to serious consequences.

RETRACTED

## 5. Conclusion

The postoperative intervention of estriol vaginal application combined with PFMT in perimenopausal patients with TH can significantly improve vaginal muscle contraction, improve the quality of sexual life, and reduce the degree of pelvic floor muscle dysfunction. Thus, PFMT combined with estriol seems promising in TH-related PFD, and its clinical applicability should be further validated in prospective multicenter studies.

## Figures and Tables

**Table 1:** General information of patients.

Items	PLMT+RT group (*n* = 49)	CT group (*n* = 46)	*t*/*χ*^2^	*P*
Age (year)	49.36 ± 4.56	48.17 ± 4.15	1.33	0.19
Number of deliveries	1.79 ± 0.54	1.81 ± 0.49	0.19	0.85
Primary diseases				
Hysteromyoma	26 (53.06%)	25 (54.35%)	0.16	0.90
Uterine adenomyoma	10 (20.41%)	9 (19.57%)	0.11	0.92
Cervical intraepithelial neoplasia	8 (16.33%)	9 (19.57%)	0.17	0.68
Abnormal uterine bleeding	5 (10.20%)	3 (6.52%)	0.08	0.78
Type of hysterectomy				
Total hysterectomy+adnexectomy	4 (8.16%)	3 (6.52%)	0.05	0.83
Total hysterectomy	2 (4.08%)	2 (4.35%)	0.04	0.76

PLMT+RT group: pelvic floor muscle training+estriol therapy group; CT group: conventional treatment group.

**Table 2:** Comparison of pelvic floor muscle tension between the two groups.

Group	Case (*n*)	Vaginal systolic pressure (cmH_2_O)		Vaginal resting pressure (cmH_2_O)	
		Before treatment	After treatment	Before treatment	After treatment
CT group	46	27.15 ± 6.59	36.17 ± 5.69^∗^	24.10 ± 4.28	30.07 ± 5.69^∗^
PFMT+ET group	49	27.47 ± 6.12	44.19 ± 5.27^∗^	24.53 ± 4.47	38.85 ± 6.21^∗^
*t*		0.127	8.989	0.045	7.936
*P*		0.789	≤0.001	0.921	≤0.001

Data was mean ± SD. ∗ indicated the paired *t*-test before and after treatment. *P* value: PFMT+ET group *vs*. CT group. PLMT+RT group: pelvic floor muscle training+estriol therapy group; CT group: conventional treatment group.

**Table 3:** Comparison of the sexual function indices of the two groups of pre- and posttreatment (scores).

Group	*n*	Pain		Satisfaction		Orgasm		Lubrication		Sexual arousal		Sexual desire		Total	
		Pre	Post	Pre	Post	Pre	Post	Pre	Post	Pre	Post	Pre	Post	Pre	Post
CT group	46	2.15 ± 1.67	4.31 ± 1.08^∗^	1.12 ± 1.29	3.45 ± 1.58^∗^	1.58 ± 0.96	2.84 ± 0.89^∗^	3.26 ± 1.63	4.01 ± 1.05^∗^	0.89 ± 0.42	3.03 ± 1.67^∗^	0.64 ± 0.25	2.85 ± 1.14^∗^	9.56 ± 4.29	19.54 ± 6.17^∗^
PFMT+ET group	49	2.20 ± 1.54	5.67 ± 1.21^∗^	1.15 ± 1.33	5.12 ± 1.14^∗^	1.49 ± 0.87	4.12 ± 1.14^∗^	3.34 ± 1.72	4.13 ± 1.14^∗^	1.85 ± 0.46	3.89 ± 1.24^∗^	0.73 ± 0.28	3.32 ± 1.20^∗^	10.03 ± 5.01	25.67 ± 5.67^∗^
*t*		0.234	6.125	0.117	5.783	0.059	6.621	0.067	0.056	0.122	5.814	0.456	5.237	0.064	7.951
*P*		0.635	≤0.001	0.851	0.001	0.842	≤0.001	0.741	0.789	0.806	0.002	0.665	0.001	0.679	≤0.001

Data was mean ± SD. ∗ indicated the paired *t*-test before and after treatment. *P* value: PFMT+ET group *vs*. CT group.

RETRACTED

**Table 4:** Comparison of the degree of pelvic floor muscle dysfunction between the two groups after the intervention.

Group	*n*	Persistent time of vaginal muscle contraction (h)		Urinary leakage in 1-hour pad test (g)		Residual urine volume (mL)		Frequency of urinary incontinence (time/d)	
		Pre	Post	Pre	Post	Pre	Post	Pre	Post
CT group	46	4.89 ± 2.13	6.25 ± 3.14^∗^	42.31 ± 8.69	22.07 ± 5.69^∗^	246.39 ± 26.58	196.67 ± 21.17^∗^	3.35 ± 0.89	2.14 ± 0.56^∗^
PFMT+ET group	49	5.02 ± 2.25	8.97 ± 4.12^∗^	44.30 ± 9.54	8.74 ± 2.14^∗^	251.19 ± 25.50	52.69 ± 8.97^∗^	3.26 ± 0.74	0.87 ± 0.42^∗^
*t*		0.246	6.374	0.157	9.531	1.023	12.207	0.039	6.573
*P*		0.641	≤0.001	0.658	≤0.001	0.962	≤0.001	0.861	≤0.001

Data was mean ± SD. ∗ indicated the paired *t*-test before and after treatment. *P* value: PFMT+ET group *vs*. CT group.

## Data Availability

The data used to support the findings of this study are available from the corresponding author upon request.
